The article "Experimental Study on Alleviating Sports Injury through Data Screening of Functional Motor Biological Images" was retracted in 2023. Reasons: signs of a paper mill; suspected computer-generated content; unreliable results or conclusions; lack of ethics approval or compliance.

# Experimental Study on Alleviating Sports Injury through Data Screening of Functional Motor Biological Images

**DOI:** 10.1155/2021/8099451

**Published:** 2021-10-06

**Authors:** Fan Rao

**Affiliations:** Physical Education Institute of Hunan Normal University, Hunan 421000, China

## Abstract

In order to better reduce sports injury, a method based on functional motion biological image data is proposed. Through performing functional motion screening test on wushu athletes, including 7 items of test, each athlete is given a score according to the test standard. This paper summarizes the mistakes and deficiencies of common movement patterns of athletes and makes different intervention plans to improve the effect of sports injury screening. The results show that, at *P* > 0.001, there was a significant difference, and the experimental group FMS total score (15.02 ± 3.7) was lower than the control group FMS total score (18.51 ± 1.45). The recognition rate of the system is higher than that of the system based on single feature, and the recognition performance is better than that of the standard SVM and KNN recognition methods. It is proved that the design of the system is feasible, reliable, and effective.

## 1. Introduction

With the rapid development of the times and economy, sports activities have reached an unprecedented level of prosperity. In various competitions, the successful holding of martial arts has been sought after and loved by many people, and the term martial arts has gradually become known to more people. Martial arts is a series of complete combinations of attack and attack moves and offensive and defensive moves. In modern times, it is a standardized sports event [1]. In form, it is a kind of exercise combining Chinese traditional martial arts with Western modern sports. In content, it has national and traditional culture, and in form, it is modern and common between China and the West [2]. With the continuous communication between Chinese and Western cultures, the continuous updating of training methods and methods, the continuous improvement of athletes' physical strength and skills, and the continuous improvement of wushu competition rules, wushu routine has formed a rich content, diverse forms, and a wide range of popular traditional sports in China. There are many martial arts movements, so it is necessary to organically combine dozens of movements arranged in advance, including the ups and downs of movements, the changes of direction, and the high intensity of difficulty, and complete them in accordance with the requirements within the specified time. In the process, there should be a distinct rhythm, the coordination of the hands, eyes, and body method in the external movement, and the unity of spirit, breath, and will in the internal, so as to achieve “power in static and method in motion,” and pay attention to the combination of internal and external and the combination of static and static throughout the whole process [3].

The article "Experimental Study on Alleviating Sports Injury through Data Screening of Functional Motor Biological Images" was retracted in 2023. Reasons: signs of a paper mill; suspected computer-generated content; unreliable results or conclusions; lack of ethics approval or compliance.

The functional action test was first proposed and applied by an American orthopaedic training expert Guy Cook and physical rehabilitation trainer Lee Brown in around 1990. Guy Cook is the leader of physical training and development in competitive sports and the pioneer of functional body training. Through long-term practice and training to develop functional body movement of the “screening” method and the basic action, the body's basic action with sports anatomy, sports biomechanics, sports physiology, and neuroscience are integrated together, through the comprehensive analysis and functional activities of final screening of action, the action is easy to operate, and the equipment requirements are not high. The stability and controllability of each action are strong, and the evaluation method is simple [4]. A comprehensive evaluation of the posture and form of the body when doing the movements such as static, dynamic, and rotating was made. It can help coaches and physical trainers to predict the weak links of athletes' body parts in advance and carry out targeted training according to the problems existing in the body, so as to achieve the goal of preventing sports injuries, enhancing the quality of various parts of the body, and prolonging the sports life. Functional motion screening was first used in 1998, and it just started to evaluate American male professional football players [5]. Before the start of the league, 50 soccer players were screened for functional movements, each player's score was recorded in detail, and the final conclusion was made. The low-scoring players were tracked throughout the season. Finally, it was found that the low-scoring players did have a risk of injury.

Charts and chart titles in the online biological literature contain rich explanatory information. If they can be effectively collected, organized, and analyzed, they will not only improve the efficiency of literature reading but also have an important significance in clinical and scientific research [6]. In recent years, a number of scholars at home and abroad have studied how to build image databases through the online biological literature, e.g., the work of Abolhasani M. In this paper, we introduce a method of automatic identification of 7 species of plankton in Jiaozhou Bay by using mathematical morphological features and Gabor texture features combined with principal component analysis and support vector machine. The experimental results show that the dimension reduction recognition based on the principal component analysis model can improve the performance of system identification; its average recognition accuracy reaches 78.5%; based on the image acquisition, image processing, and feature selection aspects for further improvement, marine plankton automatically based on the computer digital image recognition method will provide a new real-time ocean ecological environment monitoring and a fast and efficient detection platform [6]. Yamawakiet al. researched and designed the interface between generic and nongeneric modules and realized a working embedded platform. On the basis of porting the real-time operating system uCLinux to the hardware platform, this topic programmed the USB host driver to realize the communication with the image acquisition device and realized the LCD driver to display the image data and finally developed a friendly application interface call recognition algorithm with the graphics library MiniGUI [7]. The embedded system designed by Zhang et al. has realized the functions of hardware management, USB communication, and image processing through testing and has practical value. At present, the vast majority of machine vision and biological image detection are for face recognition, and there are few studies on wildlife species recognition. Biometric recognition technology mainly includes image preprocessing, feature extraction, feature selection, and classifier design. The system identifies wild bird species through convolutional neural network (CNN) and opencv convolutional neural network combined with digital image processing technology. Through the training of a large number of positive and negative samples, the characteristic files of different birds are extracted, and different images are recognized by deep learning network. The image recognition test results show that the system has high recognition efficiency and compact structure, which has certain use value [8]. Some results have been achieved. On the basis of the current research, this paper proposes a method based on functional motion biological image data screening by performing a functional motion screening test on wushu athletes, including 7 items of testing, and giving each athlete a score according to the test standards. This paper summarizes the mistakes and deficiencies of common movement patterns of athletes and makes different intervention plans to improve the effect of sports injury screening. The results show that at *P* > 0.001, there was a significant difference, and the experimental group FMS total score (15.02 ± 3.7) was lower than the control group FMS total score (18.51 ± 1.45). The recognition rate of the system is higher than that of the system based on a single feature, and the recognition performance is better than that of the standard SVM and KNN recognition methods. It is proved that the design of the system is feasible, reliable, and effective.

The article "Experimental Study on Alleviating Sports Injury through Data Screening of Functional Motor Biological Images" was retracted in 2023. Reasons: signs of a paper mill; suspected computer-generated content; unreliable results or conclusions; lack of ethics approval or compliance.

## 2. Experiment

The mode of the system platform mainly considers C/S structure (Client Server) and B/S structure (Browser Server) and combines the advantages of the two modes to build the MRI image recognition system [9]. The C/S mode is used for complex processing and security and as an interactive strong part, mainly in the image recognition input, calculation, and output. With the help of the B/S mode for the characteristics of system openness, easy maintenance, and scalability, MRI image and online literature query service is completed [10]. The development environment is Visual Studio 2005 and SQL2000, and the image feature calculation is completed by calling MATLAB 7.0-related functions [11].

The design process of the online biomedical literature MRI image recognition system mainly includes the following : (1) automatic acquisition and download of the online medical literature; (2) extracting charts and chart titles from the literature and storing them in the database; (3) the diagram containing multiple embedded images is segmented so that each embedded image is an independent image; (4) identifying the sequence number of the embedded diagram; (5) establishing the database of embedded image and embedded image annotation; (6) extracting the image features of the embedded image and the text features of the annotated pair of the embedded image; (7) labeling, classification, and recognition of block diagrams; (8) the realization, update, and improvement of the MRI image recognition system; and (9) release of the MRI image recognition system and interface with literature retrieval.

### 2.1. Research Object

During the study period, 60 wushu athletes (41 male and 19 female) were investigated for physical sports injury, and 20 athletes (165.40 + 2.22 cm in height) were selected from the sports injury group (experimental group, athletes with a history of injury within half a year) (weight 65.20 + 3.08 kg; age 21.90 + 0.86) and no injury group (control group, no injury in recent half a year, height 166.40 + 3.97 cm, weight 63.90 + 5.17 kg, and age 20.10 + 0.74 years). For details, see Table 1. In the sports injury group, there were 8 shoulder injuries, 16 lower waist injuries, 20 knee injuries, and 19 ankle injuries.

### 2.2. Research Methods

#### 2.2.1. Classification Model of the Online Biological Image Recognition System Based on the Gaussian Process

The Gaussian process is the normal stochastic process, which is a kind of universal and important stochastic process. It can be determined by means of the mean function *m*(*x*) = *E*[*f*(*x*)] and the covariance function *K*(*x*, *x*') of a random process *f*(*x*). In general, the mean function *m*(*x*) = 0 is set, and the covariance between any two different *x* values is

(1) $$\begin{array}{c} E\left[y\left(x_{m}\right)y\left(x_{n}\right)\right]=K\left(x_{m},x_{n}\right), \end{array}$$

where *K*(*x*_*m*_, *x*_*n*_)- kernel function, the kernel function with super parameter *θ* is expressed as *K*(*x*, *x*'; *θ*), and a GP is determined by the kernel type and determined hyperparameters. In this paper, three kernel functions are selected for experiments.

The article "Experimental Study on Alleviating Sports Injury through Data Screening of Functional Motor Biological Images" was retracted in 2023. Reasons: signs of a paper mill; suspected computer-generated content; unreliable results or conclusions; lack of ethics approval or compliance.

Linear kernel function:

(2) $$\begin{array}{c} \sum_{d-1}^{D}\sigma_{d}^{2}x_{d}x_{d}^{\prime }. \end{array}$$

Rational kernel:

(3) $$\begin{array}{c} {\left(1+\frac{{\left(x-x^{\prime }\right)}^{2}}{2al^{2}}\right)}^{-a}. \end{array}$$

Radial basis function:

(4) $$\begin{array}{c} \sigma_{f}.\;\exp\left(-\frac{{\left(x-x^{\prime }\right)}^{2}}{2l^{2}}\right), \end{array}$$

where *σ*, *A*, 1, and AF are all hyperparameters.

The recognition performance comparison of various methods is as follows: (1) recognition rate. The experimental results are shown in Table 2. (2) The classification results under the Gaussian radial kernel function based on different three features and the Kappa statistics of the gold standard range from 0 to 1.0. The experimental results are shown in Table 3. (3) The classification results based on different three features under the Gaussian radial kernel function are correlated with the ROC curve of the gold standard, where the cutoff point K is set to increase from 0.01 to 0.09, and the step size value is 0.01.

#### 2.2.2. The Experimental Process

60 wushu athletes (male 41 and female 19) were investigated during the research period, and 20 athletes (height 165.40 + 2.22 cm) were selected from the sports injury group (experimental group, athletes with a history of injury within half a year) (weight 65.20 + 3.08 kg; age 21.90 + 0.86) and 20 athletes without sports injury (control group, no injury in recent half a year, height 166.40 + 3.97 cm, weight 63.90 + 5.17 kg, and age 20.10 + 0.74 years); sports grade of the two groups of athletes was above that of the national level 2 athletes, and detailed information is shown in Table 1. In the sports injury group, 8 had shoulder injury, 16 had lower waist injury, 20 had knee injury, and 19 had ankle joint injury. The FMS test process is formulated according to the “Motion-Functional Movement Training System.” There are 7 tests: ① the deep-squat test, churdle-step test,② linear lunge test, ③ shoulder joint stability test (shoulder mobility test), ④ active straight leg raise test,⑤ trunk stability test,⑥ pushup test (pushup test), and ⑦ the rotary stability test, used to test the rotary stability. Each test is given a score of 0 to 3 out of a total of 21. FMS tests were performed on all athletes by the same sports medicine specialist and the total FMS score was calculated. The athlete's profile, injuries, and test scores are all entered into the Excel database. During the test, biomechanical video software was used to record the key points of athletes' bad movements. Finally, according to the results of FMS test analysis and combined with sports practice, a 4-week movement pattern correction training program was developed for problem athletes, and an injury prevention training program was developed for all athletes. After 10 weeks, the 40 athletes were given a second FMS test and interviewed again with coaches, team doctors, and athletes.

The article "Experimental Study on Alleviating Sports Injury through Data Screening of Functional Motor Biological Images" was retracted in 2023. Reasons: signs of a paper mill; suspected computer-generated content; unreliable results or conclusions; lack of ethics approval or compliance.

#### 2.2.3. Mathematical Analysis

A *T* test (SPSS18.0) was performed on the FMS test data of the injured group and the healthy group, and an Excel data radar chart was used for analysis.

## 3. Results and Analysis

The total FMS test scores of the two groups of athletes were statistically analyzed, as shown in Table 4. An independent-sample *t*-test was performed on both groups of athletes. The statistical results showed a significant difference (*P* < 0.001). The total FMS score of the experimental group (15.02 ± 3.7) was lower than that of the control group (18.51 ± 1.45).

Studies have shown that athletes with a total FMS score of less than 14 (including 14) have a higher risk of sports injury. Statistics found that 13 athletes in the experimental group scored less than 14 points, while 3 athletes in the control group scored less than 14 points. The low score data in the control group indicated that although there was a significant difference between the experimental group and the control group, and it could not be absolutely proved that the score of the experimental group athletes would be lower than 14 points, while the score of the control group athletes was higher than 14 points. The purpose of the FMS test is to quantify the quality of mobilizing motion to identify the risk of low motion quality. Through the test of the athletes with less than 14 points in the experimental group and the control group, it can be found that the athletes with less than 14 points will appear in the experimental group and the control group. This also fully shows that athletes who score less than 14 points will certainly have sports injuries, and athletes who score higher than 14 points will not necessarily be injured. The FMS test is a tool for assessing the risk of sports injuries, and a score below 14 merely indicates a high risk of sports injuries.

The article "Experimental Study on Alleviating Sports Injury through Data Screening of Functional Motor Biological Images" was retracted in 2023. Reasons: signs of a paper mill; suspected computer-generated content; unreliable results or conclusions; lack of ethics approval or compliance.

As shown in Figure 1, through the radar chart data processing of the athletes in the experimental group and the control group, the problems of the athletes in the control group were concentrated in the hurdle test and pushup test, among which the wushu athletes had problems in the stability and flexibility of the unilateral hip, knee, and ankle under the restricted condition. This also reflects that there are certain problems in the methods and means of the stable practice of one leg on the other side of the Chinese wushu athletes. The athletes in the experimental group had a series of sports injuries. More than 80% of injuries are in the lower waist, knee, and ankle joints. The knee joint injury reached 100%. Through the investigation of athletes, it is found that the knee joint injury is mainly caused by the long squatting action and the fast landing. Thus, from the FMS test, it was found that most athletes with previous sports injuries scored lower on the squat test. Squat tests are designed to assess the stability and flexibility of an athlete's shoulders, hips, knees, and ankles. This test is a comprehensive test of the overall movement pattern of the human body, which fully reflects the rationality of the sequence of joints in flexibility and stability of the human body. A score of less than 14 on this test also fully indicated that the athletes in the experimental group generally had problems with the overall movement chain. It is the existence of these problems that buries a huge risk of injury to the athletes in the training and competition of wushu.

As can be seen from Table 1, image and text feature fusion has the highest recognition rate among the classification methods based on Gaussian radial kernel function. It shows that feature fusion can improve MRI image recognition rate. From the point of view of classifiers, the classification method of radial basis kernel function based on the Gaussian process is superior to that of SVM and KNN. Kappa statistics are often used as an evaluation index to measure new methods. The larger the value is, the more stable the method will be and the higher the performance will be. As can be seen from Table 2, among the three different feature recognition methods based on image and text feature fusion, the Kappa value is above 0.8, which is the highest, indicating that the feature fusion method is better than the other two single feature-based recognition methods.

The article "Experimental Study on Alleviating Sports Injury through Data Screening of Functional Motor Biological Images" was retracted in 2023. Reasons: signs of a paper mill; suspected computer-generated content; unreliable results or conclusions; lack of ethics approval or compliance.

The larger the area enclosed by the ROC curve and the horizontal axis, the better the classification performance and stability. The area enclosed by the ROC curve and the horizontal axis based on the text and image characteristic fusion method is the largest, and its stability and performance are better than those of the single feature-based recognition method.

## 4. Corrective Training Programs and Their Effects

According to the basic model of the competitive training pyramid, the training process of athletes includes stability, flexibility, movement pattern, coordination, core stability, strength training, and power training. The study found that the wushu athletes in the experimental group had significant defects in the squat movement mode. These problems are associated with knee and ankle injuries. Therefore, a corrective training program was designed for the problems reflected in the squat test in the FMS test, as shown in Table 4.

PNF neuromuscle-facilitated drafting (PNF) and separation active stretching (AIS) were used to stretch and release the strained muscles for correction training. A mini elastic belt was used to strengthen the hip abductor muscle group and strengthen the pelvic stability. Foam axis and Bosu ball were used for hip joint flexibility training. 60 minutes of training is conducted five times a week. Finally, the problematic athletes are trained to integrate the movement chain. After 4 weeks of corrective training, the FMS test was carried out on the athletes in the experimental group. The results showed that the total average score of the second FMS test in the experimental group was 19.41, which was significantly higher than the experimental data of the pretest and the control group. The squat test scored an overall average of 3 points. On the basis of orthodontic training, shoulder joint stability training and overall functional training were added, mainly using the squat mode and kettlebell hip joint flexion and extension training. The training was for all athletes in both the experimental and control groups. The training frequency was 90 minutes three times a week.

After 10 weeks of coaching and scientific research, athletes' sports injury investigation found that the system of training, corrective and preventive, greatly reduces the number of injury. Among the 20 athletes in the experimental group, only 3 athletes had acute sports injury. During 10 weeks of training, researchers evaluated them with FMS and tested them once every 4 weeks. Every effort is made to advance the prevention window of sports injury.

## 5. Conclusions

To sum up, in the FMS test of wushu athletes, the overall performance of wushu athletes tends to be good. The FMS test can predict the risk of sports injury for wushu athletes in terms of body symmetry, balance, and flexibility, and it can be used as an indicator to evaluate the risk of sports injury. At the same time, it is a new detection tool for wushu. In order to better reduce sports injury, a method based on functional motion biological image data is proposed. Through performing a functional motion screening test on wushu athletes, including 7 items of test, each athlete is given a score according to the test standard. This paper summarizes the mistakes and deficiencies of common movement patterns of athletes and makes different intervention plans to improve the effect of sports injury screening. The results show that, at *P* < 0.001, there was a significant difference, and the experimental group FMS total score (15.02 ± 3.7) was lower than the control group FMS total score (18.51 ± 1.45). The recognition rate of the system is higher than that of the system based on single feature, and the recognition performance is better than that of the standard SVM and KNN recognition methods. The application of the FMS test can effectively detect the wrong movement patterns of wushu athletes and also provide a theoretical basis for the correction of the wrong movement patterns of wushu athletes and the application of improving their sports performance.

The article "Experimental Study on Alleviating Sports Injury through Data Screening of Functional Motor Biological Images" was retracted in 2023. Reasons: signs of a paper mill; suspected computer-generated content; unreliable results or conclusions; lack of ethics approval or compliance.

## Figures and Tables

**Figure 1:** Comparison of total FMS score data between the (a) control and (b) experimental groups.

**Table 1:** Basic information of athletes.

	Gender	Height (cm)	Weight (kg)	Age
Sports injury group	Male	165.40 + 2.22	65.20 + 3.08	21.90 + 0.86
	Female			
No sports injury group	Male	166.40 + 3.97	63.90 + 5.17	20.10 + 0.74
	Female			

**Table 2:** Recognition rates based on various methods.

Characteristics of the	GP-linear	GP-RQ	GP-RBF	KNN (*N* = 4)	SVM-RBF
Text	0.670157	0.600000	0.693194	0.700524	0.688482
Image	0.792670	0.672775	0.847539	0.826073	0843351
Text and images	0.812089	0.695812	0.895340	0.837173	0.887958

**Table 3:** Kappa values based on different feature recognition methods.

Characteristics of the	Kappa statistics
Text	0.6293
Image	0.7601
Text and images	0.8191

**Table 4:** FMS test scores.

	*n*	Minimum value	Maximum value	Average value	Standard deviation
Control group	20	12	21	18.51	1.456
Experimental group	20	8	21	15.02	3.784

## Data Availability

The data used to support the findings of this study are available from the corresponding author upon request.
